The article "Amitriptyline-Based Biodegradable PEG-PLGA Self-Assembled Nanoparticles Accelerate Cutaneous Wound Healing in Diabetic Rats" was retracted in 2024. Reason: duplicated images.

# Amitriptyline-Based Biodegradable PEG-PLGA Self-Assembled Nanoparticles Accelerate Cutaneous Wound Healing in Diabetic Rats

**DOI:** 10.3390/pharmaceutics14091792

**Published:** 2022-08-26

**Authors:** Hani Z. Asfour, Nabil A. Alhakamy, Osama A. A. Ahmed, Usama A. Fahmy, Mohamed A. El-moselhy, Waleed Y. Rizg, Adel F. Alghaith, Basma G. Eid, Ashraf B. Abdel-Naim

**Affiliations:** 1 Department of Medical Microbiology and Parasitology, Faculty of Medicine, King Abdulaziz University, Jeddah 21589, Saudi Arabia; 2 Department of Pharmaceutics, Faculty of Pharmacy, King Abdulaziz University, Jeddah 21589, Saudi Arabia; 3 Center of Excellence for Drug Research and Pharmaceutical Industries, King Abdulaziz University, Jeddah 21589, Saudi Arabia; 4 Mohamed Saeed Tamer for Pharmaceutical Industries, King Abdulaziz University, Jeddah 21589, Saudi Arabia; 5 Department of Clinical Pharmacy and Pharmacology, Ibn Sina National College for Medical Studies, Jeddah 22413, Saudi Arabia; 6 Department of Pharmacology and Toxicology, Faculty of Pharmacy, Minia University, Minia 61519, Egypt; 7 Department of Pharmaceutics, College of Pharmacy, King Saud University, Riyadh 11451, Saudi Arabia; 8 Department of Pharmacology and Toxicology, Faculty of Pharmacy, King Abdulaziz University, Jeddah 21589, Saudi Arabia

**Keywords:** diabetic wounds, amitriptyline, polymers, PEG-PLGA, nanoparticles

## Abstract

The aim of this work was to study the healing activity of amitriptyline (Amitrip) in rat diabetic wounds. A nanoformula of the drug was prepared as Amitrip-based biodegradable PEG-PLGA self-assembled nanoparticles (Amitrip-NPs) with a mean particle size of 67.4 nm. An in vivo investigation was conducted to evaluate the wound-healing process of Amitrip-NPs in streptozotocin-induced diabetic rats. Wound contraction was accelerated in rats treated with Amitrip-NPs. Histological examinations confirmed these findings, with expedited remodeling and collagen deposition in the NPs-treated animals. The formula showed anti-inflammatory activities as demonstrated by inhibition of interleukin-6 (IL-6) expression and tumor necrosis factor-α (TNF-α) expression, as well as enhanced expression of interleukin-10 (IL-10). In addition, Amitrip-NPs protected against malondialdehyde (MDA) buildup and superoxide dismutase (SOD) and glutathione peroxidase (GPx) enzymatic exhaustion. The pro-collagen activity of Amitrip-NPs was confirmed by the observed enhancement of hydroxyproline wounded skin content, upregulation of Col 1A1 mRNA expression and immune expression of collagen type IV expression. Further, Amitrip-NPs significantly increased expression transforming growth factor-β1 (TGF-β1), vascular endothelial growth factor-A (VEGF-A), platelet-derived growth factor-B (PDGF-B) and cluster of differentiation 31 (CD31). In conclusion, the developed Amitrip-NPs expedited wound healing in diabetic rats. This involves anti-inflammatory, antioxidant, pro-collagen and angiogenic activities of the prepared NPs. This opens the gate for evaluating the usefulness of other structurally related tricyclic antidepressants in diabetic wounds.

The article "Amitriptyline-Based Biodegradable PEG-PLGA Self-Assembled Nanoparticles Accelerate Cutaneous Wound Healing in Diabetic Rats" was retracted in 2024. Reason: duplicated images.

## 1. Introduction

Accumulating evidence indicates a definite link between diabetes and retarded tissue regeneration [1]. Uncontrolled diabetes can disrupt circulation, slowing blood flow and making it very difficult for the body to provide nutrients to wounds [2]. As a result, injuries may take a long time to heal or may never heal at all. Diabetic neuropathy, which affects wound healing, is another complication of diabetes. If someone is unaware of an injury, they may fail to seek care, allowing the wound to deteriorate. Infection is considerably increased by the combination of poor healing and decreased feeling in the wounded region [3]. Unfortunately, infection and development of diabetic foot ulcers are serious complications of hindered wound healing in diabetes [4]. In addition, delayed wound healing negatively affects quality of life [5]. This is in addition to the huge economic burden of non-healing wounds [6].

Amitriptyline (Amitrip) is a tricyclic antidepressant which inhibits norepinephrine and serotonin reuptake in the brain. In addition, it blocks K^+^, Na^+^ and Ca^2+^ voltage-gated ion channels [7,8]. A variety of neuropathic pain can be treated with Amitrip. Management of diabetic neuropathic pain using topical Amitrip has been previously studied [9]. The potential of antidepressants such as fluoxetine to accelerate healing of diabetic wounds has been previously reported. This was attributed to its ability to enhance TGF-β expression [10]. The role of the TGF-β family as a key player in all phases of wound healing has been reviewed [11]. Interestingly, Amitrip has also been shown to up-regulate TGF-β expression [12].

Currently, there are no satisfactory treatments for wound healing. For this reason, wound-healing medicines with varied physicochemical features can benefit from nanotechnology [13]. Biochemical properties may be easily manipulated by modifying the size and electrical charge of nanoparticles (NPs) [14]. In particular, PEG-PLGA are copolymers which are characterized by self-assembly behavior in water with amphipathic behavior [15]. Indeed, amphiphilic PEG-PLGA copolymers have attracted attention for their ability to form several forms of NPs [16]. Further, PEG-PLGA NPs are biocompatible with core architecture suitable for enclosing active substances that suffer from low water solubility, with an external hydrophilic corona that provides a shielding interface between the core and the external medium [17]. PEG-PLGA NPs are considered promising delivery systems for natural or synthetic drugs, as well as proteins such as insulin [15,17,18,19,20,21]. The aim of this work was to evaluate the ability of Amitrip-NPs formulated in an amphiphilic diblock copolymer to expedite wound healing in diabetic rats.

The article "Amitriptyline-Based Biodegradable PEG-PLGA Self-Assembled Nanoparticles Accelerate Cutaneous Wound Healing in Diabetic Rats" was retracted in 2024. Reason: duplicated images.

## 2. Materials and Methods

### 2.1. Chemicals

Amitrip, polyethylene glycol-co-poly lactide-co-glycolide (PEG-PLGA) with PEG (average molecular weight of 2000) and PLGA (average molecular number of 11,500) and lactide:glycolide 50:50, polyvinyl alcohol (PVA), hydroxypropyl methyl cellulose (HPMC) and acetone were obtained from Sigma-Aldrich (St. Louis, MO, USA).

### 2.2. Preparation of Amitrip Self-Assembled PEG-PLGA Biodegradable NPs

Amitrip-loaded PEG-PLGA NPs were prepared using the previously reported method [22,23]. Briefly, Amitrip (10% *w*/*w*) and PEG-PLGA were solubilized in acetone, and then the organic solution was added dropwise into 0.5% *w*/*v* polyvinyl alcohol (PVA) aqueous solution. The dispersion was stirred for 6 h at room temperature for complete removal of organic solvent and then subjected to probe sonication for 1 min. The produced NPs were subjected to centrifugation at 15,000× *g* for 40 min at 4 °C (Beckman Coulter Inc., Fullerton, CA, USA). The isolated NPs were re-dispersed then centrifuged twice with Milli-Q water for purification and removal of free Amitrip or excess PVA. The Amitrip-NPs were lyophilized utilizing a cryoprotectant (mannitol 5% *w*/*v*).

Amitrip-loaded hydrogel and Amitrip self-assembled PEG-PLGA-loaded hydrogel were prepared as previously described with slight modifications [24]. Briefly, raw Amitrip or its equivalent in lyophilized Amitrip self-assembled PEG-PLGA powder was dispersed in double-distilled water using a magnetic stirrer. HPMC (1.5% *w*/*w*) was added to the stirred aqueous dispersion. The formed gels were kept at 4 °C for 24 h before further use. The concentration of Amitrip or its equivalent nanoformula in the hydrogel was (2% *w*/*w*).

### 2.3. Characterization of Amitrip-NPs’ Size

The Zetasizer (Malvern, Worcestershire, UK) was utilized for measurement of the size of Amitrip-NPs. The samples were dispersed in Milli-Q water before investigation. Triplicate measurements were carried out.

### 2.4. In Vivo Study

A total of 50 male Wistar rats (200–240 g) were obtained from the Faculty of Pharmacy’s animal facility at King Abdulaziz University. The Research Ethics Committee, Faculty of Pharmacy, approved the experimental protocol (PH-1443-29). A temperature of 22 ± 2 °C was used to house the animals in 12 h day–night cycles. IP injection of streptozotocin (50 mg/kg) was used for diabetes induction, as described previously [25]. Fasting blood glucose level was checked once weekly during the course of the experiment using Accu-Chek Go (Roche, Mannheim, Germany). A range of blood glucose levels from 250 to 350 mg/dL was considered as moderate experimentally induced diabetes, and was used as the inclusion criterion for rats in the present investigation.

The article "Amitriptyline-Based Biodegradable PEG-PLGA Self-Assembled Nanoparticles Accelerate Cutaneous Wound Healing in Diabetic Rats" was retracted in 2024. Reason: duplicated images.

### 2.5. Excision Wounding and Animal Treatment

Diabetic rats were subjected to anesthesia by IP injection of ketamine (75 mg/kg)–xylazine. The dorsal area was shaved and sterilized with povidone-iodine, after which a circular excision (1 cm) was carried out [26]. A subcutaneous injection of lidocaine hydrochloride (2%) with epinephrine (1:80.000, 4.4 mg/kg) was administered near the wound area to mitigate the pain. A constant distance was used for taking the wound images with a camera (Optika, C-P5GS, Bergamo, Italy), as they were taken at their real size (1×). Wounded diabetic rats were placed in 5 groups (*n* = 10 each): the first control diabetic rats group received no treatment following induction of the wound; the second group was the negative control diabetic rats, which received only the vehicle (plain PEG-PLGA) topically on the wound every day; the third group was the diabetic rats, which received raw-Amitrip-loaded (2% *w*/*w*) gel topically; the fourth group consisted of diabetic rats, which received a topical gel loaded with Amitrip-NPs (2% Amitrip); the fifth group consisted of the positive control diabetic rats, which received Mebo^®^ ointment (Julphar, Ras Al Khaimah, UAE) on the wounded area. The ingredients of the ointment consisted of the active ingredients baicalin, berberine and β-sitosterol with beeswax as a base, as well as sesame oil. Each animal in groups 2 to 5 received the assigned treatment (0.5 g) once daily for 14 consecutive days. A dressing using a sterile gauze was placed on the wound and changed every day. Wound photographs were captured on days 0, 3, 10 and 14 after measurement of the wounded area. Wounds were treated for a total of 14 days. On day 10, 4 animals out of the group were sacrificed, as well as on day 14 (6 animals out of the group), after which skin specimens were collected from the wounds. Day 10 samples were placed in 10% neutral buffered formalin to be examined histologically. Day 14 samples were either kept in 10% neutral buffered formalin to be examined histologically and immunohistochemically, or flash-frozen to be used for biochemical and molecular studies.

The article "Amitriptyline-Based Biodegradable PEG-PLGA Self-Assembled Nanoparticles Accelerate Cutaneous Wound Healing in Diabetic Rats" was retracted in 2024. Reason: duplicated images.

### 2.6. Wound Contraction Calculation

The percentage of wound contraction was determined by (Equation (1)), taking into consideration wound diameter changes:

(1) $$\mathrm{Wound}\;\mathrm{contraction}\;\left(\%\right)=\frac{\mathrm{Wound}\;\mathrm{diameter}\;\mathrm{at}\;\mathrm{Day}\;0-\mathrm{Wound}\;\mathrm{diameter}\;\mathrm{at}\;\mathrm{Day}\;14}{\mathrm{Wound}\;\mathrm{diameter}\;\mathrm{at}\;\mathrm{Day}\;0}\times 100$$

### 2.7. Preparation of Tissue Homogenate

For preparation of tissue homogenates, injured areas were excised and cleaned with normal saline, then dried by filter paper. Skin tissue sections were kept in formalin for histopathological study. The remaining part was utilized in the biochemical study. Tissues were placed in phosphate-buffered saline (50 mM and pH 7.4) and homogenized at 4 °C in order to perform the biochemical analysis.

### 2.8. Biochemical Analysis

Homogenization of the skin samples was performed in a 10-fold amount of phosphate-buffered saline (50 mM, pH 7.4). Centrifugation was performed at 4 °C and 10,000× *g* for 15 min. The supernatant was subsequently collected and used for analysis of the parameters of oxidative stress. Kits (Biodiagnostic, Giza, Egypt), were used in the assessment of malondialdehyde (MDA, Cat.# MD2529) and superoxide dismutase (SOD, Cat.# SD2521) content and the enzymatic activity of glutathione peroxidase (GPx, Cat.# GP2524).

### 2.9. Quantitative Real-Time PCR (qRT-PCR)

A NucleoSpin^®^ kit (Macherey-Nagel GmbH, Duerin, Germany) was used to extract RNA from the skin tissue. A spectrophotometer (Dual-Wavelength, Beckman, USA) was used to determine the purity and concentration of RNA (A260/A280 ratio). A cDNA Reverse Transcription Kit (Applied Biosystems, CA, USA) was employed for reverse transcription. A Taq PCR Master Mix Kit, (Qiagen, CA, USA) along with the primers detailed in Table 1, was used for the PCR amplification reactions.

A calculation using the delta-delta Ct (ΔΔCt) method was used for relative quantitation of genes of interest [27]. GAPDH was used as the housekeeping gene. Negative controls were carried out by performing qRT-PCR runs using only the primers without the samples.

### 2.10. Histopathology

Wounded skins collected on days 7 and 14 were kept for 24 h in 10% formalin. Next, they were dehydrated using different concentrations of ethanol, cleared using xylene and paraffin-embedded [24]. Paraffinized tissue sections were sliced (5 μm thick) using a manual rotary Leica microtome, re-waxed and rehydrated. Hematoxylin and eosin (H&E) and Masson’s trichrome (MT) were used for tissue staining. Examination of the tissue sections was carried out blindly by a pathologist. Wounds were scored from “-” to “+++” according to the degree of re-epithelization, proliferation, collagen deposition and inflammatory cell infiltration, as well as progress in phases of healing.

The article "Amitriptyline-Based Biodegradable PEG-PLGA Self-Assembled Nanoparticles Accelerate Cutaneous Wound Healing in Diabetic Rats" was retracted in 2024. Reason: duplicated images.

### 2.11. Determination of IL-6, TNF-α, IL-10, TGF-β1, VEGF-A and PDGF-B, Collagen IV and CD31 Immunohistochemically

After de-paraffinization and rehydration of the tissue sections, they were boiled for 10 min in 0.1 M citrate buffer (pH 6.0). Next, sections were placed for 2 h in 5% bovine serum albumin (BSA) in Tris-buffered saline (TBS) and incubated at 4 °C with the primary antibodies anti-anti-IL-6, TNF-α, IL-10 anti-TGF-β1, anti-VEGF-A, anti-PDGF-B, collagen IV and CD31 overnight (Cat. No. ab9324, ab220210, ab33471, ab215715, ab1316, ab23914, ab6586 and ab182981, respectively, ABCAM, Cambridge, UK), all at 1 μg/mL. Anti-mouse or anti-rabbit HRP-DAB cell and tissue staining kits (Cat. No. CTS002 and CTS005, R&D Systems, Minneapolis, MN, USA) were used. After mounting, photographs of the slides were taken using a light microscope with a digital camera (Nikon SMZ 1000 and Nikon DS-Fi1, Tokyo, Japan). ImageJ software was used for image analysis (1.52a, NIH, Rockville, MD, USA). At least 3 sections per rat were included.

### 2.12. Statistical Analysis

Multiple comparisons were achieved using ANOVA, then Tukey’s post hoc tests. Statistical analyses were performed using GraphPad Prism software, version 8.0 (GraphPad, La Jolla, CA, USA). A *p*-value < 0.05 was taken as the criterion of significance.

## 3. Results

### 3.1. Preparation of Amitrip Self-Assembled PEG-PLGA Biodegradable NPs

The process of nanoprecipitation was used to create Amitrip self-assembled biodegradable PEG-PLGA NPs. The prepared Amitrip PEG-PLGA NPs showed an average particle size of less than 100 nm (67.4 ± 4.8 nm), with a polydispersity index of (0.31 ± 0.04). The biological fate of NPs in the body is primarily determined by their size.

### 3.2. Wound Healing Assessment

Figure 1A shows wound closure was fastest in diabetic rats belonging to the Amitrip-NPs group, particularly on day 10 and onwards. Figure 1B indicates that plain vehicle-treated animals did not show significant expedition of the healing rate as compared to untreated controls at all time points. On day 14, it was observed that diabetic rats’ treatment with Amitrip–nanoformula significantly enhanced the contraction of wounds (96.1%) compared to untreated control (51.3%), vehicle-treated (58.2%) and raw Amitrip (80.6%). It is worth mentioning that the Amitrip-NPs showed the most healing-accelerating action on day 14.

### 3.3. Histopathological Analysis

To further substantiate the wound healing potential of Amitrip-NPS, wounded skin was examined histologically on days 7 and 14. Skin sections stained with H&E and obtained from untreated and vehicle-treated diabetic animals on day 7 showed delayed healing, reduced re-epithelization and retarded remodeling of epidermal tissues. The wound gap was filled with necrotic collagen bundles that were heavily infiltrated by inflammatory cells, mainly neutrophils. The wound surface was covered by a thick sero-cellular crust with obvious inflammatory cells as well. However, moderate improvement was detected for raw Amitrip on days 7 and 14, as granulation tissues filling the wound gap were observed. On day 14, Amitrip-NPs animals exhibited a better grade of wound healing, with much higher collagen deposition in the formed granulation tissue associated with a marked decrease in inflammatory cells infiltration. Partial-to-complete epidermal covering was noticed in several examined sections in the Amitrip-NPs and the positive control groups. Collagen deposition (healing marker) was confirmed by Masson trichrome staining. The highest deposition of collagen in the formed granulation tissue was detected in the Amitrip-NPs group (Figure 2). These observations are semi-quantified and presented in Table 2. Amitrip-NPs had a low score of inflammatory cell infiltration with a high score of organized collagen deposition and phase II and III wound healing.

The article "Amitriptyline-Based Biodegradable PEG-PLGA Self-Assembled Nanoparticles Accelerate Cutaneous Wound Healing in Diabetic Rats" was retracted in 2024. Reason: duplicated images.

### 3.4. Effect of Amitrip-NPs on Expression of Inflammatory Biomarkers

To clarify how wounds heal following topical administration of Amitrip-NPS, immunohistochemical analysis of IL-6 and TNF-α (pro-inflammatory cytokines) as well as IL-10 (anti-inflammatory cytokine) was carried out. Figure 3 shows that treatment of diabetic rats with wounded skin with Amitrip-NPs significantly inhibited IL-6 and TNF-α expression by ~56 and ~45%, respectively, as compared to the untreated control group. The inhibition of IL-6 and TNF-α expression afforded by Amitrip-NPs was significantly lower as compared to raw Amitrip. Further, Amitrip-NPs significantly enhanced IL-10 expression by 175% as compared to the untreated control.

### 3.5. Effect of Amitrip-NPs on Biomarkers on Oxidative Status

The results in Figure 4 demonstrate that diabetic rats’ wound tissues treated with raw Amitrip or Amitrip-NPs showed lower MDA content (significantly at *p <* 0.05). Topical application of Amitrip-NPs prevented lipid peroxidation, as indicated by a significant decrease of 45% in MDA content as compared to untreated or vehicle-treated wounded skin(Figure 4A). In addition, Amitrip-NPs prevented exhaustion of SOD and GPx activity by 42% and 72% as compared to the untreated group (Figure 4B,C).

The article "Amitriptyline-Based Biodegradable PEG-PLGA Self-Assembled Nanoparticles Accelerate Cutaneous Wound Healing in Diabetic Rats" was retracted in 2024. Reason: duplicated images.

### 3.6. Effect of Amitrip-NPs on Collagen Deposition Markers

Topical application of raw Amitrip, as well as the Amitrip-NPs formulation, significantly increased (*p <* 0.05) hydroxyproline content by 100 and 171% as compared to the untreated group (Figure 5A). Similarly, both preparations significantly upregulated mRNA of Col1A1 by 230 and 331% as compared to untreated animals (Figure 5B). Amitrip-NPs treatment revealed significant enhancements in comparison to what was observed for positive-control-treated animals. Additionally, collagen type IV immune expression was significantly enhanced by Amitrip-NPs by 153% as compared to the untreated control(Figure 5C).

### 3.7. Effect of Amitrip-NPs on Expression of TGF-β1, VEGF-A and PDGF-B

The data in Figure 6 indicate that treatment of diabetic rats with Amitrip-NPs significantly enhanced TGF-β1 expression compared to the untreated, vehicle-treated and Amitrip-raw groups, by 129, 110 and 21%, respectively. In addition, VEGF-A and PDGF-B were significantly enhanced by topical application with the nanoformulation, by 140% and 137% as compared to untreated animals, respectively. It was also observed that the impact of Amitrip-NPs was comparable to the positive control group. Further, CD31 expression was significantly increased by Amitrip-NPs application, by 106% as compared to the untreated control.

## 4. Discussion

Diabetes mellitus (DM) is a common metabolic disorder due to lack of, inadequacy in or resistance to insulin. Patients are more likely to suffer foot ulcers and delayed wound healing [28]. Therefore, new and effective pharmacological interventions are required in order to positively modulate the wound-healing process, particularly in diabetic patients [10,29]. Recent years have seen increased focus on the use of nanotechnology in the pharmaceutical industry [30]. In the current study, a novel Amitrip-based biodegradable self-assembled NP of PEG-PLGA amphiphilic diblock copolymer was developed. Biocompatible nanocarriers, particularly biodegradable nanoparticles, have attracted the most attention among nanocarriers for the delivery of a variety of medications [31]. By virtue of the Amitrip-based biodegradable PEG-PLGA nano-size, it can improve how well medications pass through biological barriers [32]. Interestingly, both raw Amitrip and Amitrip-NPs proved effective at expediting wound healing in streptozotocin-diabetic rats. The prepared formula Amitrip PEG-PLGA nanoformula exhibited superior healing activities. This was proved via histological assessments which indicated the ability of the prepared formulation to inhibit inflammatory cells infiltration and increase re-epithelization and collagen deposition, hence hastening healing processes. In general, antidepressants have been reported to induce profibrotic responses via lysophosphatidic acid signaling [12]. Our data are consistent with the ability of Amitrip to enhance TGF-β release and fibrosis [33]. The positive role of the TGF-β superfamily in mediating wound healing is well-documented and has been reviewed [34]. In addition, our data are supported by the ability of the antidepressant fluoxetine to expedite wound healing in a mechanism involving stimulation of TGF-β [10].

The article "Amitriptyline-Based Biodegradable PEG-PLGA Self-Assembled Nanoparticles Accelerate Cutaneous Wound Healing in Diabetic Rats" was retracted in 2024. Reason: duplicated images.

Inflammation following tissue injury has significant roles in both normal and pathological healing. Pro-inflammatory cytokines, such as IL-6 and TNF-α, are over-produced in wounded skin [35]. Furthermore, the hypoxic environment of wounds stimulates macrophages to release several inflammatory mediators [36]. Prolonged inflammation can thus lead to delayed healing. In the current study, Amitrip exhibited anti-inflammatory activity, as evidenced by inhibition of IL-6 and TNF-α expression. This was associated with enhancement of the anti-inflammatory cytokine IL-10. Experimentally, the anti-inflammatory effects of Amitrip have been previously shown in a rat model of acetic acid-induced colitis [37]. In addition, Amitrip showed significant anti-inflammatory action in the carrageenan-induced rat paw edema model [38,39]. This is in addition to the ability of Amitrip to downregulate inflammatory responses to biomaterial in mice via inhibition of myeloperoxidase activity and the NF-κB pathway [40]. In vitro, Amitrip has been shown to inhibit nitric oxide and prostaglandin E2 production in synovial tissue cultures [41]. It is worth mentioning that Amitrip loaded in a PEG-PLGA amphiphilic diblock copolymer exhibited enhanced anti-inflammatory action. This is consistent with the ability of amphiphilic copolymers to enhance the anti-inflammatory activity of rutin, as evidenced by decreased release of IL-1β, IL-6 and TNF-α from LPS and COM-induced costimulation in thp-1 cells [42].

It has been suggested that the pathogenesis of non-healing wounds is mediated by oxidative stress [43]. In addition, therapeutic strategies targeting oxidative stress have been recommended to improve wound healing [44]. Topical application of Amitrip on the wounded skin of diabetic rats resulted in reduction in lipid peroxidation and antioxidant enzyme exhaustion. This is in harmony with several reports highlighting the antioxidant activity of Amitrip. It has been reported to ameliorate rotenone-induced Parkinson’s-like signs in rats via different mechanisms, including antioxidation [45]. Further, Amitrip has been shown to attenuate sepsis-induced brain damage via pathways involving suppression of oxidative stress [46]. In vitro, Amitrip has been reported to protect against hydrogen-peroxide-induced PC12 cell death [47]. In this study, it was also observed that PEG-PLGA-loaded Amitrip showed augmented antioxidant activity. This gains indirect support via the notion that tanshinone IIA loaded in PEG–PLGA NPs exhibited enhanced antioxidant activity and ameliorated cerebral ischemia/reperfusion injury in rats [48].

The article "Amitriptyline-Based Biodegradable PEG-PLGA Self-Assembled Nanoparticles Accelerate Cutaneous Wound Healing in Diabetic Rats" was retracted in 2024. Reason: duplicated images.

Collagen deposition, formed as a consequence of fibroblasts activation, is a critical event required to support effective wound healing [49]. Further, molecules with pro-collagen properties were suggested as potential healing agents for skin wounds [50]. The observed acceleration of wound healing afforded by Amitrip-NPs loaded in PEG-PLGA copolymer was associated with strong pro-collagen activities. This was indicated by the rise in hydroxyproline concentration, upregulation of Col 1A1 mRNA expression and enhanced expression of collagen type IV. This is supported by reports highlighting the aptitude of Amitrip to enhance experimental fibrosis as a consequence of activation of macrophage and TGF-β release [33]. Accumulating evidence indicates an important role for TGF-β in collagen formation and wound healing [34]. In this regard, our data indicate that both raw Amitrip and Amitrip-NPs loaded in PEG-PLGA copolymer significantly enhanced TGF-β expression. The NPs formula showed higher enhancing activity. TGF-β1 is an anti-inflammatory cytokine that participates in all wound-healing stages, including angiogenesis and wound closure [51]. This further supports the observed anti-inflammatory effects of Amitrip in this study. At the location of the wound, fibroblasts move during the inflammatory phase, and keratinocytes release a variety of angiogenic and growth factors [52]. In particular, angiogenesis plays a critical role in wound healing as capillary sprouts invade the wound clot, leading to the formation of a microvascular network throughout the granulation tissue [53,54]. This is in addition to the crucial role of growth factors such as TGF-β and PDGF [55]. Amitrip, in this study, enhanced the expression of VEGF-A, PDGF-β and CD31, indicating potent angiogenic and proliferative activities. This is indirectly supported by the reports showing that Amitrip induces expressions of VEGF and PDGF in primary-cultured astrocytes, [56] as well as PDGF receptors in glial cells [57]. In addition, uncontrolled diabetes has been linked to neuropathy in several pathological processes involving microvascular malfunction, polyol metabolic pathway and oxidative stress and neuroinflammation [58]. Neuropathy itself adversely affects the process of wound healing, [59] and this can be linked to decreased production of the Nerve Growth Factor [60,61]. In this regard, amitriptyline has been reported to relieve diabetic neuropathy pain [62] and possess neuroprotective effects [63,64].

The article "Amitriptyline-Based Biodegradable PEG-PLGA Self-Assembled Nanoparticles Accelerate Cutaneous Wound Healing in Diabetic Rats" was retracted in 2024. Reason: duplicated images.

## 5. Conclusions

The current study demonstrated the formulation of Amitrip-based biodegradable PEG-PLGA NPs and their potential for treating diabetic rats’ delayed healing of wounds. After 14 days of daily topical application, the developed Amitrip PEG-PLGA NPs demonstrated improved wound-healing characteristics in comparison to the raw Amitrip and a commercially available preparation. The activity of Amitrip-NPs in accelerating wound closure is attributable to their ability to decrease inflammatory cells infiltration to the wound site and increase re-epithelization. Additionally, Amitrip-NPs showed antioxidant- and collagen-enhancing activities. This was accompanied by increased protein expression of TGF-β1, PDGF-β, VEGF-A and CD31, suggesting that Amitrip-NPs further enhance proliferation and angiogenesis.

## Figures and Tables

**Figure 1:** (**A**) Diabetic rats’ wound closure for the investigated 5 groups on days 0, 3, 7, 10, 14 and 21. (**B**) Wound contraction % on day 14. Data are expressed as mean (*n* = 6) ± SD. a significantly different vs. untreated control, *p* < 0.05; b significantly different vs. vehicle-treated control, *p* < 0.05; c significantly different vs. raw Amitrip, *p* < 0.05; d significantly different vs. Amitrip-NPs, *p* < 0.05.

**Figure 2:** Histopathological effects (day 7 and 14, scale bar = 50 µm) of raw Amitrip and Amitrip-NPs on wound healing.

**Figure 3:** Effect of raw Amitrip or Amitrip-NPs on IL-6 (**upper** panel), TNF-α (**middle** panel) and IL-10 (**lower** panel) expression in diabetic rats’ wounded skin on day 14. Data are expressed as mean (*n* = 6) ± SD. a Significant vs. untreated control, *p* < 0.05; b significant vs. vehicle-treated control, *p* < 0.05; c significant vs. raw Amitrip-NPs, *p* < 0.05. Scale bar: 25 µm.

**Figure 4:** Effect of raw Amitrip or Amitrip-NPs on MDA content (**A**), SOD (**B**) and GPx (**C**) activities in diabetic rats’ wounded skin on day 14. Data are expressed as mean (*n* = 6) ± SD. a Significant vs. untreated control, *p <* 0.05; b significant vs. vehicle-treated control, *p <* 0.05; c significant vs. raw Amitrip-NPs, *p* < 0.05.

**Figure 5:** Effect of raw Amitrip or Amitrip-NPs on skin hydroxyproline content (**A**), Col 1A1 mRNA expression (**B**) and collagen type IV immune expression (**C**) in diabetic rat skin wounds of at day 14. Data are expressed as mean (*n* = 6) ± SD. a Significant vs. untreated control, *p <* 0.05; b significant vs. vehicle-treated control, *p <* 0.05; c significant vs. raw Amitrip, *p* < 0.05; d significant vs. Amitrip-NPs, *p* < 0.05. Scale bar: 25 µm.

The article "Amitriptyline-Based Biodegradable PEG-PLGA Self-Assembled Nanoparticles Accelerate Cutaneous Wound Healing in Diabetic Rats" was retracted in 2024. Reason: duplicated images.

**Figure 6:** Effect of raw Amitrip or Amitrip-NPs on TGF-β, VEGF-A (**middle**), PDGF-B and CD31 expression in diabetic rat skin wounds at day 14. Data are expressed as mean (*n* = 6) ± SD. a Significant vs. untreated control, *p <* 0.05; b significant vs. vehicle-treated control, *p* < 0.05; c significant vs. raw Amitrip, *p* < 0.05. Scale bar: 25 µm.

**Table 1:** Primer sequences used for RT-qPCR.

Gene			NCBI Reference Sequence
Col1A1	Forward	ATCAGCCCAAACCCCAAGGAGA	NM_053304.1
	Reverse	CGCAGGAAGGTCAGCTGGATAG	
GAPDH	Forward	CCATTCTTCCACCTTTGATGCT	NM_017008.4
	Reverse	TGTTGCTGTAGCCATATTCATTGT	

**Table 2:** Histological wound healing evaluation on day 14.

Group	Re-Epithelization	Fibroblast Proliferation	Collagen Deposition	Inflammatory Cell Infiltration	Phase I	Phase II	Phase III
Untreated control	-	+++	++	++	+++	++	-
Vehicle-treated	-	+++	++	++	++	++	-
Raw Amitrip	+	+	++	+	+	+++	+
Amitrip-NPs	++	+	+++	+/-	+	+++	++
Positive control	++	+	++	+	+	++	+

Wounds are scored from “-” to “+++” according to the degree of re-epithelization, proliferation, collagen deposition, inflammatory cell infiltration and progress in phases of healing.

## Data Availability

Data are contained within the article.
